The article "Differentially Expressed Genes Reveal the Biomarkers and Molecular Mechanism of Osteonecrosis" was published in 2022. Journal: J Healthc Eng.

# Differentially Expressed Genes Reveal the Biomarkers and Molecular Mechanism of Osteonecrosis

**DOI:** 10.1155/2022/8684137

**Published:** 2022-01-07

**Authors:** Huanzhi Ma, Wei Zhang, Jun Shi

**Affiliations:** Department of Orthopedic Surgery, Shandong Provincial Hospital Affiliated to Shandong First Medical University, Jinan 250021, Shandong, China

## Abstract

Osteonecrosis is one of the most refractory orthopedic diseases, which seriously threatens the health of old patients. High-throughput sequencing (HTS) and microarray analysis have confirmed as an effective way for investigating the pathological mechanism of disease. In this study, GSE7716, GSE74089, and GSE123568 were obtained from Gene Expression Omnibus (GEO) database and used to identify differentially expressed genes (DEGs) by R language. Subsequently, the DEGs were analyzed with Gene Ontology (GO) and Kyoto Encyclopedia of Genes and Genomes (KEGG) enrichment. Moreover, the protein-protein interaction (PPI) network of DEGs was analyzed by STRING database and Cytoscape. The results showed that 318 downregulated genes and 58 upregulated genes were observed in GSE7116; 690 downregulated genes and 1148 upregulated genes were screened from 34183 genes in GSE74089. The DEGs involved in progression of osteonecrosis involved inflammation, immunological rejection, and bacterial infection-related pathways. The GO enrichment showed that osteonecrosis was related with extracellular matrix, external encapsulating structure organization, skeletal system development, immune response activity, cell apoptosis, mononuclear cell differentiation, and serine/threonine kinase activity. Moreover, PPI network showed that the progression of osteonecrosis of the femoral head was related with CCND1, CDH1, ESR1, SPP1, LOX, JUN, ITGA, ABL1, and VEGF, and osteonecrosis of the jaw is related with ACTB, CXCR4, PTPRC, IL1B, CXCL8, TNF, JUN, PTGS2, FOS, and RHOA. In conclusion, this study identified the hub factors and pathways which might play important roles in progression of osteonecrosis and could be used as potential biomarkers for diagnosis and treatment of osteonecrosis.

## 1. Introduction

Osteonecrosis, characterized by eventual collapse of the femoral head, is a common bone-related disease with high incidence, especially in old people [1, 2]. The osteonecrosis of the femoral head and jaw is common typical disease of osteonecrosis, and the surgical intervention has always been used for relieving the symptom of the patients [3]. However, the pathogenic mechanism of osteonecrosis is very complex, and timely accurate diagnosis and conservative therapeutic methods may be more suitable than surgery for early patients [4]. Thus, due to limitation of special drugs, even with current intervention strategy, the outcome of the patients with osteonecrosis remains unsatisfactory. Recently, targeted drugs have been recognized as an effective way for the treatment of difficult and miscellaneous diseases. Increasing studies also confirmed that targeted therapy may also be a promising way for osteonecrosis [5].

High-throughput sequencing (HTS) is one of the most important technologies in biological research in recent years [6]. Microarray analysis based on the datasets of HTS has been confirmed as a promising and efficient strategy for the investigation of the diagnosis methods and pathogenic mechanisms of disease [7, 8]. Increasing studies have focused on illustrating the potential biomarkers and molecular mechanisms via delving global gene profiling of patients with multiple diseases ranging from epidemic to nonepidemic [9]. For osteonecrosis, several studies have also revealed the difference of the patients and normal subjects [10]. With the current biological technology, the gene profiling of the patients could be easily obtained and analyzed, and then the related strategies for the diagnosis and treatment could be developed on the basis of the body indicators of the normal persons [11].

This study attempted to (i) investigate the observed difference of expressed genes of normal and osteonecrosis patients via excavating the biological information of the chips in GEO database; (ii) identify critical factors of osteonecrosis via analyzing the gene network; (iii) and reveal the related pathological processes and signaling pathways by enrichment analysis.

## 2. Materials and Methods

### 2.1. Data Resource

The expression microarray datasets of osteonecrosis were obtained from the GEO database by R language. The microarray data of GSE74089 (GPL13497), GSE7116 (GPL570), and GSE123568 (GPL15207) were collected from GEO database in National Center for Biotechnology information (NCBI).

### 2.2. Differential Genes Analysis

For data analysis, the package of GEOquery and limma was preinstalled in R language, and then the datasets were downloaded from GEO database. For data analysis, the dataset was corrected and normalized to obtain the standardized data with high quality. After that, the difference in mRNA level of the dataset was obtained by the lmFit and eBayes function in limma package. Finally, the genes with significantly different expression (*P* < 0.05) were obtained. The corresponding *P* value of gene symbols following a *t*-test was defined as the adjusted *p* value; log2 fold change >2 and *P* < 0.05 were considered to be the cut-off criteria for differentially expressed genes (DEGs).

### 2.3. Enrichment Analysis for Related Function and Pathways of Genes

The gene enrichment analysis of Gene Ontology (GO) and Kyoto Encyclopedia of Genes and Genomes (KEGG) was performed with cluster Profiler Package of Bioconductor and David Online Database (https://david.ncifcrf.gov/). The genes in pathological group exhibiting significant difference with control (*P* < 0.05) were selected for pathway enrichment. *P* < 0.05 was set as the cut-off for enrichment analysis.

### 2.4. Protein-Protein Interaction (PPI) Network Analysis

The protein-protein interaction (PPI) network analysis of the DEGs was performed for finding key factors of the diseases. The DEGs of the datasets were analyzed with Search Tool for the Retrieval of Interacting Genes/Proteins (STRING; http://string-db.org) to obtain the data of PPI. After that, the data of the PPI were further analyzed and displayed with Cytoscape (Version 3.7.1).

## 3. Results

### 3.1. DEGs Identification in Osteonecrosis Samples

To analyze the expression difference of the normal subjects and the patients with osteonecrosis, 318 downregulated genes and 58 upregulated genes were observed in GSE7116; 690 downregulated genes and 1148 upregulated genes were screened from 34183 genes in GSE74089; 243 downregulated genes and 36 upregulated genes were screened from GSE123568 genes (Figure 1). Moreover, the top 30 genes with high differential expression in three datasets were structured with heat map (Figure 2).

### 3.2. KEGG Enrichment Analysis

To explore the regulatory pathways of the aberrant genes, the clusterProfiler, org.Hs.eg.db, and topGO were preloaded in R studio, and the KEGG enrichment was performed for analyzing the relative pathways of the DEGs of three datasets. The results showed that 47 relative pathways were obtained according to the DEGs of GSE74089, 45 pathways were obtained according to the DEGs of GSE7116, and 16 pathways were obtained according to the repetitive genes of GSE74089, GSE7116, or GSE123568 (Figures 3(a) and 3(b)). Moreover, it was also found that the pathways involved inflammatory, immune response, and infection-related pathways (Figures 3(a) and 3(b)). For repetitive genes of GSE74089, GSE7116, or GSE123568, the enriched pathways also involved the inflammation, immunological rejection, and bacterial infection (Figure 3(c)). Those proofs suggested that the progression of osteonecrosis involved inflammation, immunological rejection, and bacterial infection-related pathways.

### 3.3. GO Enrichment Analysis

To investigate the biological function of DEGs in osteonecrosis development, the DEGs of the datasets were analyzed with GO enrichment. The results showed that 164 molecular functions were found in GSE7116 and 23 molecular functions in GSE74089. Moreover, the DEGs in intersection of three datasets were also analyzed by GO enrichment, and 52 molecular functions were also found to involve the repeat genes in GSE74089 and GSE7116 (Figure 4). The GO enrichment revealed that osteonecrosis development was related with the change in extracellular matrix, external encapsulating structure organization, skeletal system development, and cellular development in GSE7116 and immune response activity, cell apoptosis, mononuclear cell differentiation, and serine/threonine kinase activity (Figure 4).

### 3.4. PPI Network Analysis

To reveal the interaction of the proteins in development of osteonecrosis, the DEGs of the GSE7116 and GSE74089 were analyzed with STRING databases and their interactive networks were structured with Cytoscape. According to the results, the networks with top three scores of GSE74089 were selected for next analysis including cluster 1 with 22 nodes and 412 edges, culster 2 with 68 nodes and 548 edges, and cluster 3 with 61 nodes and 490 edges. The networks with top three scores of GSE7116 were obtained, including cluster 1 with 24 nodes and 178 edges, cluster 2 with 14 nodes and 82 edges, and cluster 3 with 11 nodes and 50 edges. For GSE74089, CCND1, CDH1, ESR1, SPP1, LOX, JUN, ITGA, ABL1, and VEGF were hub genes which had multiple connection to other genes (Figures 5(a)–5(c)). For GSE7116, ACTB, CXCR4, PTPRC, IL1B, CXCL8, TNF, JUN, PTGS2, FOS, and RHOA were hub genes (Figures 5(d)–5(f)). Moreover, the common DEGs in GSE74089 and GSE7116 were also analyzed by PPI network, and the study showed that PTPRC and JUN were selected as hub nodes (Figure 5(g)).

## 4. Discussion

Osteonecrosis has high incidence in middle-aged and elderly age people, which seriously impacts the body functions of the patients [12, 13]. Although some studies have investigated the pathological mechanism and therapeutic methods in recent years, the systemic mechanism remains unclear. Therefore, systemic and intensive researches for key virulence factors of osteonecrosis are still necessary. In this study, the biological information of pathological samples of the subjects was obtained from the GEO database. For exploring pathological mechanism of osteonecrosis, the gene profiling datasets of the patients with osteonecrosis of the femoral head and the femoral head jaw including GSE74089, GSE123568, and GSE7116 were used to observe the expression difference of the subjects with osteonecrosis and the subjects without osteonecrosis. Moreover, a broad range of analysis strategies was performed for delving the related molecular mechanism of osteonecrosis, such as KEGG enrichment, GO enrichment, and PPI network analysis.

Osteonecrosis of the femoral head and osteonecrosis of the jaw may have certain similarity. In this study, the DEGs of GSE74089 and GSE7116 were analyzed and compared, and all the patients exhibited significant difference in some genes compared with those of the subjects without osteonecrosis, and GSE123568 including the patients steroid-induced osteonecrosis of the femoral head was also used to compare with GSE74089 and GSE7116 for revealing the key factors of the disease. The gene in the intersection of the datasets suggested that osteonecrosis of the femoral head and osteonecrosis of the jaw might involve some common core factors.

Pathway enrichment analysis is an effective strategy for biological researching, which is widely used for revealing the molecular mechanism of disease [14]. In this study, the DEGs of common factors in GSE74089 and GSE7116 were enriched in KEGG pathway and found that the development of osteonecrosis involved multiple pathway. The pathological mechanism of osteonecrosis of the femoral head and osteonecrosis of the jaw was related with the activity change of multiple pathways. Moreover, the DEGs of the patients with osteonecrosis of the femoral head or osteonecrosis of the jaw exhibited high connection with the pathways involved inflammation immune response, infection, and cancer-related pathways. Inflammation has been contributed as a major reason causing the progression of osteonecrosis. The study by Wu et al. suggested that inhibiting the TNF-*α* expression and improving the inflammatory level could effectively inhibit the development of the osteonecrosis [15]. Moreover, high levels of inflammatory factors such as IL-6 and IL-21 could also aggravate the symptom of osteonecrosis [16, 17]. The dysfunction of the immune system is the high incidence event for the patients with osteonecrosis, while the immune system sustains the normal progression of bone remodeling and tissue repair [18]. The tissues of the patients with low immune level may be susceptible to invasion by bacteria and viruses, and aberrant cells may not be timely removed by immune cells [19, 20]. The DEGs of the datasets were also analyzed with GO function enrichment. In this study, it was found that osteonecrosis development involved with the functional change of the tissues including extracellular matrix, external encapsulating structure organization, skeletal system development, and cellular development in GSE7116 and immune response activity, cell apoptosis, mononuclear cell differentiation, and serine/threonine kinase activity. Moreover, the modular functions of immune response activity were also observed in clinical data of the patients with osteonecrosis of the femoral head or osteonecrosis of the jaw.

PPI network analysis has been also used for tracking the interactions of the genes and then directly illustrated the molecular mechanism [21]. In this study, the PPI network of DEGs in the datasets was also analyzed. For osteonecrosis of the femoral head, aberrant expression of CCND1 has been also found in the patients with osteonecrosis of the femoral head induced by systemic lupus erythematosus, and ESR1 may involve the osteonecrosis development of the children with acute lymphoblastic leukemia [22, 23]. Moreover, abnormal level of VEGF was also found in gene profiling of the patients [24]. VEGF serves as key role for vascularization, and ischemia could also enhance osteonecrosis. For osteonecrosis of the jaw, it was found that TNF-*α*, ACTB, IL1B, CXCL8, PTGS2, and RHOA play hub roles in PPI network. Tumor Necrosis Factor-*α* (TNF-*α*) serves as an important inflammatory factor which could inhibit the malignant progressions of tumors and promote the inflammatory reaction of the patients [25]. Several studies have indicated that increased TNF-*α* involves the progression of osteonecrosis of the femoral head the femoral head. The study by Wu et al. has found that TNF-*α* is significantly upregulated in necrotic zone of the rats, and TNF-a-mediated alteration of M1/M2 macrophage polarization contributed to the pathogenesis of steroid-induced osteonecrosis [25]. The stability of ACTB is significantly downregulated in bone marrow-derived mesenchymal stem cells of the osteonecrosis patients [26]. Increased IL1B serves as close relationship with the progression of jaw osteonecrosis of mice, and several studies have indicated that IL1B is abnormally expressed in the serum [27]. The study by Pavlova et al. has identified CXCL8 as a potential key factor for osteonecrosis induced by Gaucher disease [28]. Chen et al. [29] has indicated that the level of PTGS2 is increasingly upregulated with the progression of osteonecrosis of the femoral head. Chen et al. have also proved that RHOA may play a hub role in progression of osteonecrosis via PPI network analysis [30]. JUN is a transcription factor, and several studies have found that c-JUN dysfunction could promote the femoral head necrosis of the rats [31]. The PPI network showed that C-JUN played a hub role in the DEGs of both patients with osteonecrosis of the femoral head or osteonecrosis of the jaw.

In conclusion, this study identified the hub factors and pathways which might play important roles in progression of osteonecrosis and could be used as potential biomarkers for diagnosis and treatment of osteonecrosis.

## Figures and Tables

**Figure 1:** Volcano plots of differentially expressed genes between patients with osteonecrosis and related controls. Red nodes are upregulation and blue nodes are downregulation. (a) The expressed genes of GSE7116. (b) The expressed genes of GSE74089. (c) The expressed genes of GSE123568.

**Figure 2:** Heat maps of differentially expressed genes between patients and related controls. Orange represents upregulation and blue represents downregulation. (a) The expressed genes of GSE7116. (b) The expressed genes of GSE74089. (c) The expressed genes of GSE123568.

**Figure 3:** The pathways involved in osteonecrosis development. (a) Module gene KEGG enrichment analysis of GSE74089. (b) Module gene KEGG enrichment analysis of GSE7116. (c) Venn diagram of GSE74089, GSE7116, and GSE123568. The larger the size, the more significant the proportion of the gene.

**Figure 4:** The modular functions involved in osteonecrosis development. (a) Module gene GO enrichment analysis of GSE74089. (b) Module gene GO enrichment analysis of GSE7116. The larger the size, the more significant the proportion of the gene.

**Figure 5:** The PPI network of DEGs in osteonecrosis. (a–c) The PPI network of GSE74089. (d–f) The PPI network of GSE7116. (g) The PPI network of the common DEGs of GSE74089 and GSE7116.

## Data Availability

The data used to support the findings of this study are available on reasonable request from the corresponding author.
